# Modeling the Ranked Antenatal Care Visits Using Optimized Partial Least Square Regression

**DOI:** 10.1155/2022/2868885

**Published:** 2022-03-14

**Authors:** Maryam Sadiq, Alanazi Talal Abdulrahman, Randa Alharbi, Dalia Kamal Fathi Alnagar, Syed Masroor Anwar

**Affiliations:** ^1^Department of Statistics, University of Azad Jammu and Kashmir, Muzaffarabad, Pakistan; ^2^Department of Mathematics, College of Science, University of Hail, Saudi Arabia; ^3^Department of Statistics, University of Tabuk, Saudi Arabia; ^4^Department of Statistics, Omdurman Islamic University, Sudan

## Abstract

The frequency and timing of antenatal care visits are observed to be the significant factors of infant and maternal morbidity and mortality. The present research is conducted to determine the risk factors of reduced antenatal care visits using an optimized partial least square regression model. A data set collected during 2017-2018 by Pakistan Demographic and Health Surveys is used for modeling purposes. The partial least square regression model coupled with rank correlation measures are introduced for improved performance to address ranked response. The proposed models included PLS*ρ*_*s*_, PLS*τ*_*A*_, PLS*τ*_*B*_, PLS*τ*_*C*_, PLS _*D*_, PLS*τ*_*GK*_, PLS _*G*_, and PLS _*U*_. Three filter-based factor selection methods are executed, and leave-one-out cross-validation by linear discriminant analysis is measured on predicted scores of all models. Finally, the Monte Carlo simulation method with 10 iterations of repeated sampling for optimization of validation performance is applied to select the optimum model. The standard and proposed models are executed over simulated and real data sets for efficiency comparison. The PLS*ρ*_*s*_ is found to be the most appropriate proposed method to model the observed ranked data set of antenatal care visits based on validation performance. The optimal model selected 29 influential factors of inadequate use of antenatal care. The important factors of reduced antenatal care visits included women's educational status, wealth index, total children ever born, husband's education level, domestic violence, and history of cesarean section. The findings recommended that partial least square regression algorithms coupled with rank correlation coefficients provide more efficient estimates of ranked data in the presence of multicollinearity.

## 1. Introduction

Pakistan sets targets to minimize the maternal mortality ratio (MMR) to 140 per 100,000 live births by 2015 by increasing skilled birth attendants and improving access to reproductive health care as the fifth Millennium Development Goal (MDG) for improving maternal health suggested. The MDG progress assessment reported that Pakistan was not close to attaining the target in 2015. Recently, Pakistan has endorsed the Sustainable Development Goals (SDGs), committing to decrease the MMR to 70 per 100,000 live births by 2030 by increasing skilled birth attendance, facilitation to modern contraception, and extending coverage of health workers. The Government of Pakistan took initiatives and made good progress in maternal health indicators during the last decade, and a significant decline was reported in MMR from 276 to 178 [1, 2]. Pregnancy-related morbidity and mortality can be reduced by improving access and facilitation to maternal health care services. At least four antenatal care visits (ANC) are recommended to skilled personnel to avoid any pregnancy-related complication [3]. Nearly 12% Pakistani women reported no ANC throughout their pregnancy, 36% have less than four visits, and 52% claimed four or more visits [1]. Several studies have assessed the significant influential factors of antenatal care attendance in Pakistan without considering the frequency of ANC [4, 5]. Poisson regression, negative binomial regression, zero-inflated, and hurdle regression models have been commonly used to model the count of ANC visits [6, 7]. Binary logistic regression and a multinomial logistic regression model are also found to study the use and ranks of ANC visits [5, 8]. Advancements in health research generate public health data having many covariates, where some or all may be correlated. Several studies have been conducted to identify influential factors of different public health concerns using multiple statistical tools and techniques [9–13]. The partial least square (PLS) regression model has been the concern of interest as a statistical method for modeling data having multicollinearity during the last few decades. A variety of modified PLS algorithms have been introduced for superior model performance [14]. Most PLS algorithms model continuous factors, and a few are specifically designed for categorical framework but no specific algorithm is projected to address the ranked data. To fill the gap of obtaining the optimal model for the ranked response variable, modified PLS algorithms based on ranked correlation loading weights are introduced. The main motivation of the present study is to propose the modified PLS algorithms to particularly address the ranked response factor in the presence of multicollinearity. To improve the PLS regression model, eight algorithms based on rank correlation measures including Spearman's rank correlation coefficient, Kendall's *τ*_*A*_ rank correlation coefficient. Kendall's *τ*_*B*_ rank correlation coefficient, the Stuart-Kendall *τ*_*C*_ rank correlation coefficient, Somers' delta (*D*), Goodman-Kruskal's tau *τ*_*GK*_, Goodman-Kruskal's gamma (*G*), and Thiel's *U* correlation coefficient are proposed in this study. To the best of our knowledge, no previous research has considered multicollinear covariates in modeling the ranking of ANC visits of Pakistani women. Thus, the objectives of this study are twofold: (i) to develop a regression model for the ranked response covering the issue of multicollinearity and (ii) to determine the risk factors for inadequate use of antenatal care. This study introduced eight novel PLS algorithms addressing the concern of multicollinearity for a ranked response which is never discussed earlier. The proposed and standard algorithms are executed on a real-life application of ANC data for comparison purposes. These algorithms will facilitate users to obtain more efficient models than the standard PLS approaches for specifically ranked data. Regarding the clinical importance of this study, the influential selected variables of ANC will help maximize the chances for a normal pregnancy by providing priority interventions, increasing coverage, and improving health quality. The novel contribution of this study included:

- eight new PLS algorithms based on rank correlation loading weights are proposed to address rank response
- the significant factors of ANC utilization of Pakistani women are identified

## 2. Methodology

### 2.1. Data Set

The data acquired from Pakistan demographic and health survey (PDHS) 2017-2018 for Baluchistan is used for the present study. A total of 943 observations (women) with 43 factors are included in the analysis. The frequency of ANC is considered the ordinal response factor (*y*) which is ranked as inadequate (0-3 visits), intermediate (4-7 visits), and adequate (8-9 visits).

### 2.2. Partial Least Square Regression (PLSR)

Consider the regression model *y* = *α* + *Zβ* + *ε*, where *α* and *β* are the unknown regression parameters and *ε* is the error term. Let *Z*_(*n*, *p*)_ is the matrix of explanatory variables and is assumed to be linearly related with the response *y*_(*n*, 1)_ and suppose some *C* (where *C* ≤ *p*) to represent the number of components for prediction. Then, for *c* = 1, ⋯, *C*, the general algorithm executes as

1. The loading weights are *w*_*c*_ = *Z*′_*c*−1_*y*_*c*−1_
2. The score vector is *t*_*c*_ = *Z*_*c*−1_*w*_*c*_
3. Evaluate *Z*-loadings (*P*_*c*_) and *Y*-loadings (*q*_*c*_) by *p*_*c*_ = *Z*′_*c*−1_*t*_*c*_/*t*′_*c*_*t*_*c*_ and *q*_*c*_ = *y*′_*c*−1_*t*_*c*_/*t*′_*c*_*t*_*c*_, respectively
4. Deflate *Z*_*c*−1_ and *y*_*c*−1_ by *Z*_*c*_ = *Z*_*c*−1_ − *t*_*c*_*p*′_*c*_ and *y*_*c*_ = *y*_*c*−1_ − *t*_*c*_*q*_*c*_
5. Repeat the algorithm, if *c* < *C*

Consider that *W*, *S*, *P*, and *q* are the matrices/vectors to compile the loading weights, scores, *Z*-loadings, and *Y*-loadings computed at each iteration of the algorithm, respectively. The regression estimators of the PLSR model are computed by $\hat{\beta }=W{\left(P^{\prime }W\right)}^{-1}q$ and $\hat{\alpha }=\bar{y}-\bar{Z}\hat{B}$ [15]. The general steps of standard PLSR are presented in Figure 1.

The standard PLS is designed for continuous dependent variable *y* but if the response is measured on a rank scale then this standard method may not work well. The most important phase of the PLS algorithm is to compute loading weight having the ability to choose significant factors. Loading weights compute the correlation between the dependent variable and predictors. If the data set is ranked then Spearman's rank correlation coefficient, Kendall's *τ*_*A*_ rank correlation coefficient, Kendall's *τ*_*B*_ rank correlation coefficient, the Stuart-Kendall *τ*_*C*_ rank correlation coefficient, Somers' delta (d), Goodman-Kruskal's tau *τ*_*GK*_, Goodman-Kruskal's Gamma (*G*), and Thiel's *U* correlation coefficient are the recommended measures of rank correlation. These measures of association are used to compute the loading weights of the PLS algorithm. The modified loading weights of PLSR are visually displayed in Figure 2.

#### 2.2.1. PLS*ρ*_*s*_

Spearman's rank correlation coefficient or Spearman's *ρ* (*ρ*_*s*_) [16] is a nonparametric measure of rank correlation using a monotonic function. It is used to compute the weights of as

(1) $$\begin{array}{c} w_{\rho_{s}}=1-\frac{6\sum d_{i}^{2}}{n\left(n^{2}-1\right)}, \end{array}$$

where *d*_*i*_ denotes the difference between the two ranks of each observation and *n* is the number of observations and the modified PLSR algorithm is referred to as PLS*ρ*_*s*_.

#### 2.2.2. PLS*τ*_*A*_

The Kendall rank correlation coefficient or Kendall's *τ* coefficient is a measure of rank correlation. The tau-*A* (*τ*_*A*_) will not make any adjustment for ties [17]. It is used to define the PLS loading weights as

(2) $$\begin{array}{c} w_{\tau_{A}}=\frac{n_{c}-n_{d}}{n_{0}}, \end{array}$$

where *n*_*c*_ is the number of concordant pairs, *n*_*d*_ is the number of discordant pairs, and *n*_0_ = *n*(*n* − 1)/2, and the modified algorithm is named as PLS*τ*_*A*_.

#### 2.2.3. PLS*τ*_*B*_

Kendall's tau-*B* makes adjustments for ties [18]. The PLS loading weights are altered by using *τ*_*B*_ as

(3) $$\begin{array}{c} w_{\tau_{B}}=\frac{n_{c}-n_{d}}{\sqrt{\left(n_{0}-n_{1}\right)\left(n_{0}-n_{2}\right)}}, \end{array}$$

where *n*_1_ = ∑_*i*_*t*_*i*_(*t*_*i*_ − 1), *n*_2_ = ∑_*j*_*u*_*j*_(*u*_*j*_ − 1), *t*_*i*_ is the number of tied value in the *i*^th^ group of ties and *t*_*j*_ is the number of tied value in the *j*^th^ group of ties and the proposed model is termed as PLS*τ*_*B*_.

#### 2.2.4. PLS*τ*_*C*_

The Stuart-Kendall (tau-c) is more suitable for contingency tables [19]. The *τ*_*C*_ replaced the weights of PLS as follows:

(4) $$\begin{array}{c} w_{\tau_{C}}=\frac{2\left(n_{c}-n_{d}\right)}{n^{2}\left(\left(m-1\right)/m\right)} \end{array}$$

where *m* is the minimun number among rows and coulmns, and the modified PLSR algorithm is called PLS*τ*_*C*_.

#### 2.2.5. PLS _*D*_

The PLS loading weights based on Somers' delta(*D*) [20] of variable *Y* with respect to variable *Z* are defined as

(5) $$\begin{array}{c} w_{D}=\frac{\tau \left(Z,Y\right)}{\tau \left(Z,Z\right)}. \end{array}$$

Kendall's tau *τ* is symmetric, whereas Somers' *D* is asymmetric in *Z* and *Y*, and the model is named as PLS _*D*_.

#### 2.2.6. PLS*τ*_*GK*_

Goodman-Kruskal's tau *τ*_*GK*_ [21] is integrated as PLS loading weights as

(6) $$\begin{array}{c} w_{\tau_{GK}}=\frac{2\left(n_{c}-n_{d}\right)}{n_{0}}, \end{array}$$

and the modified algorithm is called PLS*τ*_*GK*_.

#### 2.2.7. PLS _*G*_

The estimate of Goodman-Kruskal's gamma (*G*) [21] is used as loading weights of PLS

(7) $$\begin{array}{c} w_{G}=\frac{n_{c}-n_{r}}{n_{c}+n_{r}}, \end{array}$$

where *n*_*c*_ is the number of concordant pairs and *n*_*r*_ is the number of reversed pairs. Goodman-Kruskal's gamma drop ties, and the PLSR model is named as PLS _*G*_.

#### 2.2.8. PLS _*U*_

Thiel's *U* correlation coefficient or uncertainty coefficient [22] altered the PLS loading weights as

(8) $$\begin{array}{c} w_{U}=\frac{H\left(Z\right)-H\left(Z\;|\;Y\right)}{H\left(Z\right)}, \end{array}$$

where *H*(*Z*) represents the entropy of a single distribution and *H*(*Z* | *Y*) represents the conditional entropy, and the modified PLSR algorithm is referred to as PLS _*U*_.

### 2.3. Filter-Based Factor Selection Methods

Several variable selection methods integrated with PLSR have been introduced. The following are considered here.

#### 2.3.1. The Loading Weight (LW)

The loading weights *w*_*j*_ are used to measure of importance of predictors and are defined as [23].

(9) $$\begin{array}{c} \text{LW}=\left|\frac{w_{a,j}}{\max\left(w_{a}\right)}\right|. \end{array}$$

#### 2.3.2. The Regression Coefficients (RC)

The regression coefficient estimates are computed as [23]

(10) $$\begin{array}{c} \text{RC}=W{\left(P^{\prime }W\right)}^{-1}q. \end{array}$$

#### 2.3.3. Significance Multivariate Correlation (SMC)

The significance multivariate correlation measure is used to reduce the effect of irrelevant predictors and enhance the influence of significant variables included in the model. The SMC [23] is computed as

(11) $$\begin{array}{c} \text{SMC}=\frac{\text{MeanSquareRegression}}{\text{MeanSquareResidual}}. \end{array}$$

## 3. Results

Initially, the PLS models with modified loading weights are executed for simulated data set for ranked variables. A sample of size 1000 with 100 predictors is generated. The response variable and 50% predictors are generated over 3 ranks, and the remaining explanatory variables are distributed over 4 ranks.

Spearman's coefficient, Kendall's coefficient-*A*, Kendall's coefficient-*B*, Stuart-Kendall's, Somers' delta, Goodman-Kruskal's tau, Goodman-Kruskal's gamma, and Thiel's *U* coefficient are used as loading weights of the PLS algorithm to fit oversimulated data set to observe the variation in performance of standard and proposed models based on Akaike information criterion (AIC).

Figure 3 showed the efficiency of models established by AIC and indicated that PLSR algorithms with modified loading weights have higher efficiency (lower mean AIC) compared to standard PLSR for a ranked response. The PLSR model with *τ*_*GK*_ as modified loading weight showed optimum performance compared to eight other models without integrating any variable selection method. All other proposed models also evidenced higher efficiency compared to standard PLSR. Figures 4 and 5 also demonstrated the higher accuracy of proposed models compared to standard PLSR algorithm integrated with LW and SMC variable selection methods. Both figures depicted that PLS*τ*_*GK*_ and PLS _*U*_ have optimum performance compared to all other models. The standard and modified models are also executed over the real data set of ANC for comparison of accuracy. The data set of ANC visits had 43 predictors sampled over 943 samples (mothers). The Spearman rank correlation coefficient is used to examine the multicollinearity in the data. The correlogram map measured strong correlation among 16 covariates while intermediate correlation among several other predictors is observed and shown in Figure 6. The existence of multicollinearity recommends the applicability of PLSR to deal ranked data with multicollinearity.

The frequency of ANC is classified into three ranks as inadequate, intermediate, and adequate. The ratio of 70 : 30 is used to randomly split data into training and testing sets, respectively. Initially, PLSR integrated with rank correlation coefficients as loading weights is executed. The Spearman's coefficient, Kendall'scoefficient-*A*, Kendall's coefficient-*B*, Stuart-Kendall's, Somers' delta, Goodman-Kruskal's tau, Goodman-Kruskal's gamma, and Thiel's *U* coefficient are used to modify loading weights. Then, three filter-based factor selection methods are performed on each of the nine PLSR models. Leave-one-out cross-validation by linear discriminant analysis is measured on predicted scores of all 27 models. Finally, the Monte Carlo simulation method is used with 10 iterations of repeated sampling for optimization of validation performance. The standard PLSR is compared with the PLSR integrated with Spearman's coefficient (PLS*ρ*_*s*_), PLSR integrated with Kendall's coefficient-*A* (PLS*τ*_*A*_), PLSR integrated with Kendall's coefficient-*B* (PLS*τ*_*B*_), PLSR integrated with the Stuart-Kendall (PLS*τ*_*C*_), PLSR integrated with Somers' delta (PLS _*D*_), PLSR integrated with Goodman-Kruskal's tau (PLS*τ*_*GK*_), PLSR integrated with Goodman-Kruskal's gamma (PLS _*G*_), and PLSR integrated with Thiel's *U* coefficient (PLS _*U*_).

Figure 7 showed the comparison of validation performance of standard PLSR and eight proposed PLSR models integrated with correlation coefficients without considering any variable selection method. These results depicted that PLS*ρ*_*s*_ and PLS _*D*_ have optimum performance compared to standard PLSR and other proposed PLSR models for the observed data of ANC visits. The PLS *τ*_*A*_ and PLS*τ*_*GK*_ also have relatively higher accuracy than standard PLSR. In Figure 8, the loading weight factor selection method is incorporated with each PLSR model. The inclusion of the variable selection method enhanced the overall performance of standard and modified PLSR models. The results showed that PLS*τ*_*A*_ and PLS*τ*_*B*_ are more efficient in terms of optimization accuracy compared to standard and modified PLS models. A similar pattern of performance for PLS*ρ*_*s*_ and PLS*τ*_*C*_ is observed compared to standard PLSR. Four other proposed PLSR models integrated with rank correlation coefficients showed slightly lower accuracy compared to standard PLSR.

Figure 9 established performance comparison of the PLSR model based on the RC factor selection method. The results demonstrated that compared to PLSR, the six proposed methods including PLS*ρ*_*s*_, PLS*τ*_*A*_, PLS*τ*_*B*_, PLS*τ*_*C*_, PLS _*D*_, and PLS _*U*_ featured incremental performance after accounting RC selection method. Two other proposed methods PLS*τ*_*GK*_ and PLS _*G*_ demonstrated approximately identical efficiency as standard PLSR. Standard and modified PLSR models embedded with the SMC factor selection method are compared in Figure 10 in terms of validation accuracy. The two proposed PLSR models including PLS*ρ*_*s*_ and PLS*τ*_*C*_ evidenced higher accuracy than standard PLSR. The other four modified models including PLS*τ*_*A*_, PLS _*D*_, PLS _*G*_, and PLS _*U*_ measured analogous accuracy as PLSR.

Comparison based on validation accuracy supported that PLS*ρ*_*s*_ is found to be the most appropriate proposed method to model the observed ranked data set of ANC. Figure 7 represented the optimal performance of PLS*ρ*_*s*_ compared to all other models without considering any variable selection method. Integrated with RC factor selection methods, the proposed PLS*ρ*_*s*_ showed higher efficiency compared to standard PLS visualized in Figure 9. Moreover, PLS*ρ*_*s*_ established the highest optimization accuracy of nearly 78% among all other methods in 10 combined with the SMC factor selection method. Based on this evidence, PLS*ρ*_*s*_ featured with the SMC method is finally picked for the selection of influential factors of ANC. For extraction of influential factors of ANC, PLS*ρ*_*s*_ coupled with SMC is executed and estimates of 29 variables are presented in Table 1 with regression estimates.

## 4. Discussion

To examine the significant predictors associated with ANC, sample data obtained from PDHS (2017-2018) is used. The occurrence of multicollinearity pointed to the application of PLS being a popular substitute for the standard regression model. Data is randomly divided into testing and training sets. Eight PLS algorithms established on rank correlation coefficients are introduced to address particularly the ranked response and compared with the standard PLS model to prove the improved efficiency in model building. The proposed models include Spearman's coefficient (PLS*ρ*_*s*_), PLSR integrated with Kendall's coefficient-*A* (PLS*τ*_*A*_), PLSR integrated with Kendall's coefficient-*B* (PLS*τ*_*B*_), PLSR integrated with the Stuart-Kendall (PLS*τ*_*C*_), PLSR integrated with Somers' delta (PLS _*D*_), PLSR integrated with Goodman-Kruskal's tau (PLS*τ*_*GK*_), PLSR integrated with Goodman-Kruskal's Gamma (PLS _*G*_), and PLSR integrated with Thiel's *U* coefficient (PLS _*U*_).

Furthermore, three variable selection methods are integrated with standard and modified PLS algorithms to estimate the accuracy to examine the variation in the performance of modified and standard PLS models with and without variable selection methods. The variable selection methods, namely, loading weights, regression coefficients, and significance multivariate correlation are considered here. The validation performance is computed for 10 iterations to examine the efficiency of nine PLS models integrated with variable selection methods.

Comparison based on validation performance supported that PLS*ρ*_*s*_ is found to be the most appropriate proposed method to model the observed ranked data set of ANC. Figure 7 represented the optimal performance of PLS*ρ*_*s*_ compared to all other models without considering any variable selection method. Integrated with RC factor selection methods, the proposed PLS*ρ*_*s*_ showed higher efficiency compared to standard PLS visualized in Figure 9. Moreover, PLS*ρ*_*s*_ established the highest optimization accuracy of nearly 78% among all other methods in 10 combined with the SMC factor selection method. Based on this evidence, PLS*ρ*_*s*_ featured with the SMC method is finally picked for the selection of influential factors of ANC.

Regarding validation accuracy, very important and interesting facts are observed about the comparison of efficiency for ranked data. Primarily, PLS*ρ*_*s*_ and PLS _*D*_ have optimum performance compared to standard PLSR and other proposed models without considering any factor selection method. For the observed data set, the PLS*τ*_*A*_ and PLS*τ*_*B*_ combined with the LW variable selection method are found to be more efficient in terms of optimization accuracy compared to standard and modified PLS models. Integrated with RC method for variable selection, the PLS*ρ*_*s*_, PLS*τ*_*A*_, PLS*τ*_*B*_, PLS*τ*_*C*_, PLS _*D*_, and PLS _*U*_ featured incremental performance compared to standard PLS. The PLS*τ*_*GK*_ and PLS _*G*_ are found to exhibit approximately similar efficiency as standard PLSR. The PLS*ρ*_*s*_ and PLS*τ*_*C*_ embedded with the SMC factor selection method evidenced optimum accuracy compared to standard PLS. Considering all validation comparisons, it is noticed that the modified models integrated with rank correlation coefficient exhibit higher efficiency for ranked data set of ANC compared to the standard PLS algorithm. The PLS*ρ*_*s*_ coupled with SMC is suggested for modeling the ANC ranked data and 29 influential factors are observed to discriminate the ANC ranks. The proposed algorithms for rank response will facilitate researchers to address the regression models more efficiently even in the presence of multicollinearity in different fields of research. Since the rank response is specifically addressed rarely, the findings of this study offer new, potentially useful information for this ranked population. In the future, these algorithms may be integrated with other variable selection methods to observe the efficiency. Also, the proposed study can be extended for neutrosophic statistics [9]. The main limitation of this study is the small number of predictors as every possible factor was not available for the target population and also the interaction effects are not included.

## 5. Conclusion

Proposed PLS algorithms integrated with rank correlation coefficients are observed to be a better option with regard to model efficiency and variable selection of ranked simulated and real data sets. This suggests that these rank measure-based PLS algorithms provide models with superior potential. The PLS*ρ*_*s*_ coupled with SMC identified the significant predictors of ANC using the optimized model for the observed data. The modified PLS models have the ability to address multicollinear ranked data more effectively. Regarding the clinical importance of this study, the influential selected variables of ANC will help maximize the chances for a normal pregnancy by providing priority interventions, increasing coverage, and improving health quality.

## Figures and Tables

**Figure 1:** Standard PLS algorithm.

**Figure 2:** Modified loading weights of PLS.

**Figure 3:** The AIC performance of PLSR models based on rank correlation coefficients' oversimulated data without considering any variable selection method is presented.

**Figure 4:** The AIC performance of PLSR models based on rank correlation coefficients' oversimulated data integrated with LW variable selection method is presented.

**Figure 5:** The AIC performance of PLSR models based on rank correlation coefficients' oversimulated data integrated with SMC variable selection method is presented.

**Figure 6:** Correlogram by Spearman rank correlation matrix is presented. Color intensity and the size of the circle are proportional to the strength of the correlation among covariates.

**Figure 7:** The validation accuracy of PLSR models based on rank correlation coefficients including Spearman's correlation coefficient (Rho), Kendall coefficient-*A* (tau-*A*), Kendall coefficient-*B* (tau-*B*), Stuart-Kendall (tau-*C*), Somers' delta (Delta), Goodman-Kruskal's tau (GKTau), Goodman-Kruskal's gamma (GKGamma), and Thiel's *U* coefficient (UCoef) models is presented.

**Figure 8:** The validation accuracy of PLSR models based on rank correlation coefficients integrated with LW factor selection method is presented.

**Figure 9:** The validation accuracy of PLSR models based on rank correlation coefficients integrated with the RC factor selection method is presented.

**Figure 10:** The validation accuracy of PLSR models based on rank correlation coefficients integrated with SMC factor selection method is presented.

**Table 1:** Regression coefficient estimates of influential factors for PLS*ρ*_*s*_ coupled with SMC.

Factor	Coefficient
Age of women	0.010
Type of residence	-0.036
Women's educational level	0.061
Source of drinking water	-0.036
Age of household head	0.023
Frequency of watching television	0.022
Wealth index	0.052
Total children ever born	0.048
Births in last five years	0.016
Number of living children	-0.037
Ever had a terminated pregnancy	-0.034
Visited health facility last 12 months	0.021
Previous birth a caesarean section	0.047
Getting medical help for self: getting permission to go	-0.030
Getting medical help for self: getting money needed for treatment	0.045
Getting medical help for self: distance to health facility	0.021
Heard of tuberculosis	-0.023
Husband's education level	0.040
Respondent's occupation	0.037
Husband's age	-0.017
Beating justified if wife neglects the children	-0.012
Beating justified if wife argues with husband	-0.049
Beating justified if wife refuses to have sex with husband	0.042
Sex of child	0.015
Number of pregnancy losses	0.035
Blood relationship with husband	-0.035
Had a say in choosing the husband	0.026
Ever heard of hepatitis B or C	-0.028
Receive any cash/kind benefit from Benazir Income Support Program	-0.024

## Data Availability

Data is available at https://dhsprogram.com/data/.
